The article "Magnetic Resonance Imaging Image Feature Analysis Algorithm under Convolutional Neural Network in the Diagnosis and Risk Stratification of Prostate Cancer" was published in 2021. Journal: J Healthc Eng.

# Magnetic Resonance Imaging Image Feature Analysis Algorithm under Convolutional Neural Network in the Diagnosis and Risk Stratification of Prostate Cancer

**DOI:** 10.1155/2021/1034661

**Published:** 2021-11-27

**Authors:** Weijun Gao, Peibo Zhang, Hui Wang, Pengfei Tuo, Zhiqing Li

**Affiliations:** ^1^Department of Urology Surgery, 215 Hospital of Shaanxi Nuclear Industry, Xianyang 712000, Shaanxi, China; ^2^Department of Urology, Affiliated Hospital of Yan'an University, Yan'an 716000, Shaanxi, China; ^3^Department of Urology, Yan'an Hospital of Traditional Chinese Medicine, Yan'an 716000, Shaanxi, China

## Abstract

This work aimed to explore the accuracy of magnetic resonance imaging (MRI) images based on the convolutional neural network (CNN) algorithm in the diagnosis of prostate cancer patients and tumor risk grading. A total of 89 patients with prostate cancer and benign prostatic hyperplasia diagnosed by MRI examination and pathological examination in hospital were selected as the research objects in this study (they passed the exclusion criteria). The MRI images of these patients were collected in two groups and divided into two groups before and after treatment according to whether the CNN algorithm was used to process them. The number of diagnosed diseases and the number of cases of risk level inferred based on the tumor grading were compared to observe which group was closer to the diagnosis of pathological biopsy. Through comparative analysis, compared with the positive rate of pathological diagnosis (44%), the positive rate after the treatment of the CNN algorithm (42%) was more similar to that before the treatment (34%), and the comparison was statistically marked (*P* < 0.05). In terms of risk stratification, the grading results after treatment (37 cases) were closer to the results of pathological grading (39 cases) than those before treatment (30 cases), and the comparison was statistically obvious (*P* < 0.05). In addition, it was obvious that the MRT images would be clearer after treatment through the observation of the MRT images before and after treatment. In conclusion, MRI image segmentation algorithm based on CNN was more accurate in the diagnosis and risk stratification of prostate cancer than routine MRI. According to the evaluation of Dice similarity coefficient (DSC) and Hausdorff I distance (HD), the CNN segmentation method used in this study was more perfect than other segmentation methods.

## 1. Introduction

Prostate malignant tumor (prostate cancer) is the one with the highest incidence among all types of tumors of the male urinary system, ranking 6th in China and around the world [1], and it is most common in middle-aged and elderly men [2]. For different regions and races, the difference in the mortality and incidence of prostate cancer is very clear [3]. In recent years, in terms of the incidence of male cancers, prostate cancer has become the second most common cancer after lung cancer [4]. Whether the diagnosis of this disease is accurate is related to the good or bad prognosis of prostate cancer treatment [5]. At this stage, prostate-specific antigen (PSA) is the primary screening method, but its accuracy is not high. However, a biopsy of puncture samples is harmful to patients and lays a heavy economic burden on them [6]. According to research, magnetic resonance imaging (MRI) has a higher value, among which nuclear MRI (NMRI) can be called a meaningful enhancement of imaging technology in the field of medicine, and has occupied a very important position in the field of medical imaging. Moreover, MRI imaging is free of ionizing radiation and is harmless to the human body, which is convenient for women during pregnancy. With high contrast, MRI can be used for multidirectional and multiparameter imaging, which can diagnose diseases—to determine the location, nature of the disease, and the stage of the tumor and to judge the curative effect—to evaluate the effectiveness of the treatment plan [7]. Furthermore, MRI is globally recognized as the preferred method for the early diagnosis and staging of prostate cancer.

The article "Magnetic Resonance Imaging Image Feature Analysis Algorithm under Convolutional Neural Network in the Diagnosis and Risk Stratification of Prostate Cancer" was published in 2021. Journal: J Healthc Eng.

The prostate is composed of central glands and marginal glands, and the structure of the prostate of different individuals is quite different. The key to diagnosing prostate cancer is to accurately and quickly find the boundary of the prostate and separate it from other tissues [8]. However, it is difficult to segment the entire prostate gland with traditional MRI technology, and the operation process is also very cumbersome and complicated. Deep learning, especially the rapid development of artificial intelligence, promotes the methods of computer vision and medical image processing. The use of deep learning neural network algorithm makes the image segmentation technology more and more mature and fast and can also simplify the image processing process.

Kearney et al. [9] proposed a deeply supervised CNN model to segment prostate MRI images. This model can effectively detect the prostate area and add a new layer of deep supervision. However, the individual differences of the prostate, the interference of surrounding tissues, and imaging artifacts still have a great impact on the segmentation of MRI [10].

According to the above content, there are still some shortcomings, although deep learning neural network has been applied to clinical diagnosis and treatment. The patients with prostate cancer were taken as the research objects in this study, and the segmentation processing of their MRI images with the convolutional neural network (CNN) algorithm was optimized to evaluate whether the MRI image analysis algorithms based on CNN were accurate in the diagnosis and risk assessment of prostate cancer. Therefore, a certain reference basis for the diagnosis and treatment of prostate cancer patients could be provided.

The article "Magnetic Resonance Imaging Image Feature Analysis Algorithm under Convolutional Neural Network in the Diagnosis and Risk Stratification of Prostate Cancer" was published in 2021. Journal: J Healthc Eng.

## 2. Materials and Methods

### 2.1. Research Objects and Grouping

The prostate cancer patients and benign prostatic hyperplasia patients, who were diagnosed by MRI and pathological examinations in hospital from September 2018 to March 2020, were selected as the research objects. A total of 89 cases passed the exclusion criteria. The patients were all male and 39–74 years old, with an average age of 49 years. The MRI images of these patients were collected in two groups and enrolled into a pretreatment group and a posttreatment group. The number of research cases in both groups was 89, and the results were compared with the known pathological biopsy results. The process had been approved by the ethics committee of the hospital, and all the research objects included in this study signed the informed consent forms.

The inclusion and exclusion criteria of research objects were as follows. The criteria for inclusion were defined to include patients who did not receive the surgical treatment or prostate biopsy before MRI examinations, had the multisequence and multidirectional MRI scanning, and had no other malignant tumor lesions. The criteria for exclusion were defined to include patients who underwent the biopsy of diseased tissue before MRI, received the relevant treatment before the MRI examinations, had the prosthesis in the detected part, had the moving artifacts in the images, had the incomplete MRI images, and had no pathological confirmation after MRI.

### 2.2. Examination Method

All patients were scanned at the pubic symphysis with the same scanning instrument. Each patient should relax, exhale normally, and take the supine position. The scanning position and parameters are shown in Figure 1. The prostate MRI scan sequence included oblique axis position T2-weighted imaging (T2WI) + Fs (scanning level perpendicular to the long axis of the prostate), oblique axis position T2WI (scanning level perpendicular to the long axis of the prostate), oblique coronal position T2WI + Fs (scanning level parallel to the long axis of the prostate), sagittal T2WI + Fs, oblique axis T1WI + Fs (scanning level perpendicular to the long axis of the prostate), and oblique axis T1WI (scanning level perpendicular to the long axis of the prostate).

The article "Magnetic Resonance Imaging Image Feature Analysis Algorithm under Convolutional Neural Network in the Diagnosis and Risk Stratification of Prostate Cancer" was published in 2021. Journal: J Healthc Eng.

### 2.3. Establishment of Prostate Segmentation Model Based on the Convolutional Neural Network Algorithm

CNN is mainly composed of a convolutional layer, a pooling layer, a fully connected layer, and a deconvolutional layer [11]. The *h* layer is set as the convolutional layer, and then the feature map of the MRI image was input in the *h* − 1 layer, which can be expressed as follows:

(1) $$\begin{array}{c} A\left(h,p\right)=\sum_{b=1}^{B}Y^{\left(h,p,b\right)}⊗Z^{\left(h-1,b\right)}+l^{\left(h,p\right)}, \end{array}$$

where *Y*^(*h*, *p*, *b*)^ represents the convolution kernel, *l*^(*h*, *p*)^ expresses the bias, *b* stands for the number of feature maps, and *Z* means the target image.

To improve the network's ability to express data features, a nonlinear activation function is proposed [12]. In this study, ReLu was selected as the activation function, which was commonly used and had a high rate. Its expression equation is equation (2), and the corresponding derivative function's expression equation is equation (3). Among them, *x* represents the number of samples.

(2) $$\begin{array}{c} f\left(x\right)=\max\left(0,x\right), \end{array}$$

(3) $$\begin{array}{c} f^{\prime }\left(x\right)=\left\{\begin{array}{cc} x, & x>0,\\ 0, & x\leq 0. \end{array}\right. \end{array}$$

*G* was supposed as the MRI image of the prostate. All pixels in image *G* were expressed by *S*, and the collection form was (*s*_1_, *s*_2_,…, *s*_*n*_). The image was divided into those parts that were denoted by *U*, and the expression was (*u*_1_, *u*_2_,…, *u*_*n*_). The prostate includes the central gland and the marginal gland, which should be distinguished from the surrounding tissues. Thus, it can be divided into three parts: the central gland, marginal gland, and surrounding tissues; namely, *U* = 3. Then, for pixel *s*_*n*_ of the *j*-th channel, the probability of corresponding output *u*_*j*_ was as follows:

(4) $$\begin{array}{c} p\left(s_{n}=u_{j}\right)=\frac{1}{E}\exp\left[v\left(u_{j}\right)\right]. \end{array}$$

In equation (4), *v*(*u*_*j*_) refers to the value of *u*_*j*_, *E* is the regularization term, and the predicted value *y*_*n*_ obtained by *s*_*n*_ could be expressed as *y*_*n*_=arg max[*p*(*s*_*n*_=*u*_*j*_)]. Besides, the corresponding loss function can be expressed as follows:

(5) $$\begin{array}{c} L=-\frac{1}{cd}\sum_{n}\sum_{j}y_{nj}\ln\left[p\left(s_{n}=u_{j}\right)\right]. \end{array}$$

Batch normalization (BN), a neural network optimization method, can reduce the difficulty of learning, thereby increasing the speed of model practice. This method refers to a step of preprocessing in advance when processing each layer to standardize the data [13]. In this study, this method was employed to improve the algorithm based on CNN. In addition, the expression of BN is as follows:

(6) $$\begin{array}{c} {\bar{X}}^{i}=\frac{X^{\left(i\right)}-Y\left[X^{i}\right]}{\sqrt{\text{Var}\left[X^{\left(i\right)}\right]}}. \end{array}$$

In equation (6), *Y*[*X*^*i*^] is the mean of each group of samples *X*^(*i*)^ and Var[*X*^(*i*)^] was the variance, but there was a problem with the expression. Thus, Vaughan introduced new parameters *χ* and *λ*. Then, the expression of the new BN is presented in the three following equations:

(7) $$\begin{array}{c} Q^{i}=\chi^{\left(i\right)}{\bar{X}}^{\left(i\right)}+\lambda^{\left(i\right)}, \end{array}$$

(8) $$\begin{array}{c} \chi^{\left(i\right)}=\sqrt{\text{Var}\left[X^{\left(i\right)}\right]},\lambda^{\left(i\right)}=Y\left[X^{i}\right], \end{array}$$

(9) $$\begin{array}{c} Y=\frac{\chi }{\sqrt{\text{Var}\left[X\right]+\gamma }}.X+\left(\lambda -\frac{\chi Y\left(X\right)}{\sqrt{\text{Var}\left[X\right]+\gamma }}\right). \end{array}$$

BN belongs to a single layer and is usually placed behind the base layer of the roll and in front of the activation function.

The article "Magnetic Resonance Imaging Image Feature Analysis Algorithm under Convolutional Neural Network in the Diagnosis and Risk Stratification of Prostate Cancer" was published in 2021. Journal: J Healthc Eng.

The operation of the pooling layer-based semantic segmentation (PSSNET) is shown in the following equation:

(10) $$\begin{array}{c} FP_{i}^{h+1}=\frac{1}{k_{p}^{2}}F_{i}^{h+1}*KP. \end{array}$$

In equation (10), *F*_*i*_^*h*+1^ represents the *i*-th convolution kernel in the *L* + 1-th layer, *FP*_*i*_^*h*+1^ stands for the *i*-th feature map in the *L*-th layer, *k*_*p*_^2^ is the size of the pooling window, and *KP* expresses a matrix of all 1.

Besides, the processing process is shown in Figure 2. First, the convolution method is employed to extract the image features, and the deconvolution method is used for segmentation after the extraction is completed.

### 2.4. MRI Image Quality Evaluation Indexes and Standards

(1) The quality of MRI images processed based on the deep CNN technology was evaluated, and the evaluation indexes were as follows:
  The two following methods were adopted to determine how to evaluate whether the results of the prostate segmentation algorithm based on the CNN algorithm were ideal and effective compared with the expert segmentation of the region after the completion of MRI image processing. First, the Dice similarity coefficient (DSC) in this study referred to the degree of overlap between the area segmented by doctors and the area segmented by PSSNET, and its calculation equation is as follows:
    (11) $$\begin{array}{c} \text{DSC}=\frac{2\left|M\cap N\right|}{\left|M\right|+\left|N\right|}. \end{array}$$
  In the above equation, *M* stands for the standard region value segmented by the doctor, and *N* refers to the result region segmented by the CNN model. According to the above equation, the range of DSC was taken as [0, 1]. When the minimum value was taken as 0, *M* and *N* did not overlap. On the contrary, *M* and *N* were perfectly overlapped if the maximum value was 1. This showed that the larger the DSC value, the higher the coincidence degree of *MN* and the better the segmentation result, and vice versa.
  Second, the Hausdorff distance (HD) represented the maximum range of mismatch between the two sets of numbers, which was used to evaluate the similarity of the two sets of numbers. The points in the MRI images of the *M* group could be set as *M*={*m*_1_, *m*_2_, *m*_3_,…, *m*_*x*_}, and the points in the *N* group were *N*={*n*_1_, *n*_2_, *n*_3_,…, *n*_*x*_}, as shown in the three following equations:
    (12) $$\begin{array}{c} \text{HD}\left(M,N\right)=\max\left(h\left(M,N\right),h\left(M,N\right)\right), \end{array}$$
    (13) $$\begin{array}{c} h\left(M,N\right)=\max\left(m\in M\right)\min\left(n\in N\right)\left\|m-n\right\|, \end{array}$$
    (14) $$\begin{array}{c} h\left(M,N\right)=\max\left(n\in N\right)\min\left(m\in M\right)\left\|n-m\right\|. \end{array}$$
  The smaller the HD value, the higher the similarity and the higher the mid-overlap of the image. In other words, the result was the most ideal when *M* = *N*.
(2) The segmentation effect of the PSSNET method in the CNN was compared with that of Deeplabv3 + and Pixenet that was explored by previous researchers.
(3) The characteristics of routine MRI images and CNN-based MRI images were compared to observe the sharpness and resolution of the images.
(4) The positive rate of MRI diagnosis based on the CNN was compared with that of pathological detection based on the test results of pathological tissue biopsy. The MRI images based on the CNN were divided into a low-risk group, a medium-risk group, and a high-risk group using Gleason scoring criteria, as shown in Table 1, as well as PSA and clinical stage of tumor [14], and the results were compared with pathological grading results.

The article "Magnetic Resonance Imaging Image Feature Analysis Algorithm under Convolutional Neural Network in the Diagnosis and Risk Stratification of Prostate Cancer" was published in 2021. Journal: J Healthc Eng.

### 2.5. Statistical Methods

The test data processing was carried out using SPSS 19.0 statistical software. The measurement data were expressed as the mean ± standard deviation ($\bar{x}$ ± *s*), the *t*-test was used for the comparison of the means in each group, the count data were represented by percentage (%), and the *χ*^2^ test was adopted. In addition, *P* < 0.05 meant that the difference was statistically substantial.

## 3. Results

### 3.1. Comparison on MRI Image Evaluation Based on Convolutional Neural Network Algorithm and Other Methods

The MRI image segmentation area processed by the CNN segmentation method was compared and analyzed with the target area marked by professional doctors, and the data were brought into two evaluation accuracy standards, namely, the equations of DSC and HD. The obtained results were DSC = 0.916 and HD = 0.819. According to the content of Section 2.4, the value of HD was smaller if the value of DSC was larger, and then the result of image processing was better and the accuracy was higher. Single data could hardly explain whether this result was good or bad. In order to determine whether PSSNet was effective in processing MRI images, the same data were brought into other existing segmentation methods. The results obtained are shown in Figure 3, suggesting that the processing results of PSSNet were the most effective compared with those of other methods.

### 3.2. Routine MRI Imaging Features of Patients with Prostate Cancer and Prostate Hyperplasia

The MRI images of various diseases of the prostate were very similar to the MRI images of prostate cancer, so it was difficult to distinguish between ordinary ultrasound and other examinations. The normal MRI images of the prostate are presented in Figure 4. The shape and size of the prostate in the images were all similar to a flat chestnut. The upper end was wide, the lower end was tapered, and the back of the body was relatively flat. The longitudinal diameter was about 3 cm, the transverse diameter was about 4 cm, and the front and back diameters were about 2 cm.  Figure 5 shows the comparison of MRI images between prostate cancer and benign prostatic hyperplasia. Since the lesion area and normal tissues of the prostate under T1WI scanning showed a low-medium signal, it was difficult to distinguish. Thus, it was the result of scanning under the T2WI sequence. Although the difference in the signal of the MRI images could be observed, it was not very clear. The range of the lesion was generally discernible, but the boundaries were blurred, which brought some interference to the differential diagnosis of the disease.

### 3.3. CNN-Based MRI Image Features of Patients with Prostate Cancer and Other Prostate Diseases

Compared with Figure 4, the imaging in Figure 5 was clearer and can distinguish between the diseased area of prostate disease and the normal tissue by using the signal with obvious difference in height.  Figure 6 reveals that the lesion ranges of prostate cancer and hyperplasia were very similar to the signal. They were both low signal areas and invaded the surrounding normal gland tissue. Such a clear image would improve the accuracy of the doctor's diagnosis of the disease, but it was still difficult to diagnose the benign and malignant lesions.

The article "Magnetic Resonance Imaging Image Feature Analysis Algorithm under Convolutional Neural Network in the Diagnosis and Risk Stratification of Prostate Cancer" was published in 2021. Journal: J Healthc Eng.

### 3.4. Comparison on the Diagnosis Results and Risk Stratification of MRI Images Based on CNN and the Detection Results of Pathological Tissue Biopsy

#### 3.4.1. Comparison on Diagnosis Results

Taking the results of pathological biopsy as the standard, 39 cases of prostate cancer and 50 cases of prostate hyperplasia were obtained. What is more, the comparison with the results obtained by observing MRI images is shown in Table 2. The positive rate of pathological biopsy was 44%, the positive rate of MRI image results before processing was 34%, and the positive rate of MRI results after processing was 42%. Through the comparison, it is indicated that the CNN-processed MRI results were more similar to the pathological biopsy results, and the comparison was statistically obvious (*P* < 0.05). Thus, it is suggested that MRI images based on CNN could diagnose diseases more accurately than routine MRI, as shown in Figure 7.

#### 3.4.2. Comparison on the Risk Classification of Prostate Cancer Diagnosis Results

Assessment of the risk of prostate cancer for patients can help determine the best treatment plan.

In this study, MRI and pathological testing were employed to stage tumors, and the risk of patients with prostate cancer was assessed by combining with Gleason score and PSA. Table 2 shows the number of prostate cancer cases diagnosed under different testing methods. Therefore, the cancer patients under pathological and MRI detection were 39/30/37, and the staging results are shown in Table 3. The accuracy rate of tumor staging obtained by tissue biopsy was higher. By comparison, it was found that the results of MRI images after processing of the number of cases in each risk grade were closer, and the comparison was statistically significant (*P* < 0.05). It is also shown that MRI images based on CNN were more accurate in tumor staging of prostate cancer than routine MRI (Figures 8 and 9).

## 4. Discussion

Based on the data analysis of the results obtained in this study, MRI images based on CNN were more accurate in the diagnosis of prostate diseases than routine MRI images. The application of deep learning artificial intelligence in the medical field is very extensive, and the combination of deep learning neural networks and medical imaging is becoming more and more inseparable. The research on the application of MRI imaging technology combined with artificial intelligence in the diagnosis and treatment of various diseases has become a global hot spot.

The CNN investigated in this study has also been researched by many experts. Among them, Long et al. [15] proposed for the first time and perfectly combined fully CNN (FCNN) with image segmentation to create a new path for image segmentation. With the advancement of deep learning, Li et al. [16] combined neural network segmentation algorithms with medical image segmentation and won first place in the cell image segmentation competition of the Medical Image Computing and Computer-Assisted Intervention Society (MICCAI) at that time. In the field of prostate image segmentation, Jin et al. [17] proposed and applied a three-dimensional neural network to the segmentation of prostate MRI for the first time. Bustin et al. [18] applied the three-dimensional neural network formed by the long-short-jumping connection method to the MRI image of the prostate, which made the MRI segmentation on the three-dimensional interface more accurate. Tian et al. [19] optimized the neural network for prostate segmentation and achieved good results. In this study, the CNN segmentation technology was applied to segment MRI images of prostate patients, which also achieved good results. The results obtained were DSC = 0.916 and HD = 0.819. Fehri et al. [20] developed a two-way recursive neural network that can use contextual features to transform prostate blocks into data sets for processing and used it in prostate segmentation. Greer et al. [21] studied the sensitivity and specificity of several imaging experts from different levels of various hospitals to changes in the condition, determined whether their observations were consistent, and then used computer-assisted diagnosis (CAD) to diagnose the same MRI images again. It was concluded that the MRI detection assisted by CAD had good consistency and sensitivity, but the specificity was not good enough. Varghese et al. [22] combined imaging and machine learning (ML) and cross-checked the accuracy of multiple ML algorithms for the detection of clinically significant prostate cancer. Besides, the subcore-based support vector machine (SVM) method had the best accuracy, up to 92%. The CNN technology combined with MRI images in this study was more accurate in diagnosing prostate cancer. The positive rate of pathological biopsy was 44%, and the positive rate of MRI results after processing reached 42%. The positive rate of posttreatment MRI was 42%, and the positive rate of pretreatment routine MRI was 34%.

The article "Magnetic Resonance Imaging Image Feature Analysis Algorithm under Convolutional Neural Network in the Diagnosis and Risk Stratification of Prostate Cancer" was published in 2021. Journal: J Healthc Eng.

Based on the above research information, artificial intelligence based on deep learning was gradually being combined with medical imaging technology, and, after continuous research and improvement by professional technicians, good research results were achieved, and it was gradually applied to clinical diagnosis and treatment.

## 5. Conclusion

The results of pathological biopsy diagnosis were taken as the standard in this study, and there was a comparison of the diagnostic results of routine MRI images and CNN segmentation algorithm-processed MRI images. Through the analysis of the data and results obtained from this study, it was concluded that the MRI image segmentation algorithm based on CNN was more accurate in the diagnosis of prostate cancer and the risk stratification of prostate cancer than routine MRI. The DSC and HD standards were used to evaluate the excellence of this segmentation method. After comparing the results obtained by other segmentation methods, the results of this method were relatively the best. Through research, the MRI image segmentation method based on CNN had more effective diagnostic value for the diagnosis of prostate diseases, thereby providing a more effective reference basis for clinical diagnosis and treatment. However, due to the single acquisition range of the sample and lack of representativeness, the further improvements will be made in subsequent research. It is hoped that the network algorithm of deep learning can provide a good auxiliary effect for the detection of clinical diseases.

## Figures and Tables

**Figure 1:** MRI scanning process.

**Figure 2:** Process of segmentation of prostate based on CNN algorithm.

**Figure 3:** Comparison on DSC and HD results of different MRI segmentation methods.

**Figure 4:** MRI images of normal prostate: (a) the coronal section and (b) the horizontal section.

**Figure 5:** Comparison on MRI images of prostate cancer and benign prostatic hyperplasia. (a) Prostate cancer. (b) Hyperplasia of prostate.

**Figure 6:** Comparison on MRI images of prostate cancer and prostate hyperplasia after optimized treatment. (a) Prostate cancer. (b) Hyperplasia of prostate.

**Figure 7:** Comparison on the MRI results before and after image processing and the results of pathological biopsy: (a) before processing; (b) after processing.

**Figure 8:** Comparison on risk levels of MRI before image processing and pathological examination.

**Figure 9:** Comparison on the risk levels between MRI after image processing and pathological examination.

**Table 1:** Gleason grading criteria.

Grading	Manifestation
Gleason1	Cancer tissue is extremely rare. Its borders are very clear, it grows expansively, and it hardly invades the matrix; the carcinomas are simple, usually round, and moderately sized and are packed together; the cytoplasm of cancer cells closely resembles that of benign epithelial cells.
Gleason2	Cancer tissue is rare, which mostly occurs in the transitional area of the prostate. The tumor boundary is not very clear, and the carcinomas are separated by the stroma. They are simple, round, different in size, and irregular in shape and are loosely arranged together.
Gleason3	Cancer tissue is the most common, which mostly occurs in the peripheral area of the prostate. Its most important feature is invasive growth, the carcinomas are of different sizes and shapes, nucleoli are large and red, and the cytoplasm is mostly alkaline staining.
Gleason4	The cancer tissue is poorly differentiated and grows infiltrating; the carcinomas are irregularly fused to form tiny papillary or sieve-shaped, large and red nucleoli; the cytoplasm can be alkaline or gray.
Gleason5	The cancer tissue is very poorly differentiated. The border can be regularly round or irregular, accompanied by invasive growth; the growth form is sheet-like single cell type or acne-like carcinoma type, accompanied by necrosis; cancer cells have large nuclei and large and red nucleoli; cytoplasmic staining may vary.

The article "Magnetic Resonance Imaging Image Feature Analysis Algorithm under Convolutional Neural Network in the Diagnosis and Risk Stratification of Prostate Cancer" was published in 2021. Journal: J Healthc Eng.

**Table 2:** The detection results of prostate through pathological biopsy and MRI.

Detection methods		Symptoms	
		Cancer	Hyperplasia
Results of histopathological examination		39	50
Results of histopathological MRI examination	Before processing	30	59
	After processing	37	52

**Table 3:** Results of prostate cancer risk stratification under different test methods.

		Low-risk group	Medium-risk group	High-risk group
Pathological examination		14^*∗*^	17^*∗*^	8^*∗*^
MRI	Before processing	20	9	10
	After processing	15^*∗*^	16^*∗*^	8^*∗*^

^*∗*^Tthe difference was statistically marked (*P* < 0.05).

## Data Availability

The data used to support the findings of this study are available from the corresponding author upon request.
